# Long non-coding RNA H19 induces hippocampal neuronal apoptosis *via* Wnt signaling in a streptozotocin-induced rat model of diabetes mellitus

This article has been retracted.

**DOI:** 10.18632/oncotarget.17472

**Published:** 2017-04-27

**Authors:** Yu-Hao Zhao, Tie-Feng Ji, Qi Luo, Jin-Lu Yu

**Affiliations:** ^1^ Department of Neurosurgery, The First Hospital of Jilin University, Changchun, P.R. China; ^2^ Department of Radiology, The First Hospital of Jilin University, Changchun, P.R. China

**Keywords:** long non-coding RNA H19, hippocampal neurons, diabetes mellitus, Wnt signaling pathway, streptozotocin, Pathology Section

## Abstract

Defects in hippocampal synaptic plasticity and disorders of memory and learning are the central nervous system complications of diabetes mellitus (DM). Here, we used a streptozotocin-induced rat DM model to investigate the effects of long non-coding RNA H19 (lncRNA H19) on learning and memory and apoptosis of hippocampal neurons, and the involvement of the Wnt signaling. Our data demonstrate that lncRNA H19 is highly expressed in rats with DM. Over-expression of lncRNA H19 increased positioning navigation latency in DM rats and decreased duration of space exploration. lncRNA H19 over-expression also increased hippocampal neuronal apoptosis and expression of Wnt3, β-catenin, TCF-1, Bax, caspase-8 and caspase-3. By contrast, expression of GSK-3β and Bcl-2 was suppressed in DM rats over-expressing lncRNA H19. These results suggest that lncRNA H19 induces hippocampal neuronal apoptosis *via* Wnt signaling, and that inhibition of lncRNA H19 may serve as a promising novel target for the treatment of cognitive decline in patients with DM.

## INTRODUCTION

Diabetes mellitus (DM) is a group of metabolic diseases characterized by hyperglycemia, insulin resistance, and/or insulin deficiency [1]. The chronic hyperglycemia of DM is associated with long-term dysfunction, damage, and multiple organ failure, particularly kidney, eye, heart, nerve, and blood vessel dysfunction [2]. In addition, DM adversely affects the brain, which undergoes changes that may increase the risk of cognitive decline [3]. Animal models with DM exhibit biochemical and behavioral deficits, particularly in the hippocampus, a brain region important for memory and learning [4]. For example, DM rats spend less time exploring novel objects, supporting a deficit of memory processing [5]. In addition, DM rats have decreased locomotor activity and higher immobility during a forced swim test [5].

Long non-coding RNAs (lncRNAs) are essential for higher cognitive abilities and brain development, and are involved in psychiatric diseases, providing tissue- and activity-specific epigenetic and transcriptional regulation [6]. *H19* gene is a paternally imprinted gene located near the telomeric region of chromosome 11p15.5, an area frequently involved in adult and pediatric tumors [7]. Almost 98% of the “junk” DNA is transcribed to non-coding RNAs (ncRNAs), including short ncRNAs and lncRNAs [8]. The human *H19* gene encodes a 2.3 kb long, polyadenylated and spliced ncRNA that is vital in embryonal growth control [9]. The lncRNA H19 has been associated with the regulation of human tumor growth [10] and activation of the Wnt signaling pathway [11]. In addition, Wnt signaling is an essential regulator of adult hippocampal neurogenesis, and Wnt protein regulates adult hippocampal function [12]. A dynamic gradient of Wnt signaling pathway can regulate cellular specification in the hippocampus and initiation of neurogenesis in the mammalian cortex [13]. The modules transducing Wnt signaling are well conserved throughout evolution, and β-catenin plays a vital role in the canonical Wnt signaling [14].

In this study, we hypothesized that lncRNA H19 might regulate apoptosis of hippocampal neurons *via* the Wnt signaling. Using a rat DM model, we investigated the impact of lncRNA H19 on learning and memory, apoptosis of hippocampal neurons, and involvement of the Wnt signaling.

## RESULTS

### Expression of lncRNA H19 in the hippocampal tissues

The expression of lncRNA H19 in the hippocampus tissues was analyzed by qRT-PCR. Compared to the normal group, the expression of lncRNA H19 was significantly increased in the empty vector model, NC, and over-expressed lncRNA H19 groups (all *P* < 0.05), while it was decreased in the lncRNA H19-shRNA group (*P* < 0.05). There was no significant difference between the lncRNA H19-shRNA and normal groups (*P* > 0.05). The expression of lncRNA H19 in the over-expressed lncRNA H19 group was higher than in the model and empty vector groups (all *P* < 0.05), and there was no statistically significant difference between these two groups (*P* > 0.05). The expression of lncRNA H19 in the lncRNA H19-shRNA group was decreased compared to the model and NC groups (*P* < 0.05), and there was no statistically significant difference between these two groups (*P* > 0.05) (Figure 1).

**Figure 1:** Expressions of Lnc RNA H19 in hippocampal tissues of rats in each group measured by qRT-PCR Notes: *, *P* < 0.05 as compared with the normal group; #, *P* < 0.05 as compared with the model group; &, *P* < 0.05 as compared with the empty vector group; $, *P* < 0.05 as compared to the NC group; NC = negative control; qRT-PCR = quantitative real-time plymerace chain reaction.

### Whole gene methylation in rat models of the normal and model groups

Compared to the normal group, hippocampal tissues of DM rats showed hypomethylation in the model group (Figure 2) (*P* < 0.01). In the model group, the methylation in H19 promoter region was lower than in the normal and NC groups (all *P* < 0.01).

**Figure 2:** The expression of whole genome methylation in rat model of the hippocampal tissues and the expression of methylation from H19 promoter region of LncRNA H19 Notes: **A.**, Elisa detected the expression of whole genome methylation of the hippocampal tissues; **B.**,**C.**, the expression of methylation from H19 promoter region of LncRNA H19; ** indicated *P* < 0.01 as compared to the normal group; LncRNA = long non-coding RNA.

### Blood glucose levels and body weight in DM rats

In the normal group, there was no significant difference in basal blood glucose levels, blood glucose levels after rat modeling, and random blood glucose levels at 12 weeks (*P* > 0.05). The basal blood glucose levels in the individual groups were not significantly different (all *P* > 0.05). Compared to the normal group, the blood glucose level after modeling in each group significantly increased (all *P* < 0.05). At 12 weeks, the blood glucose levels in the empty vector, over-expressed lncRNA H19, model, and NC groups increased (all *P* < 0.05). There was no significant difference in the lncRNA H19-shRNA and normal groups (*P* > 0.05). Compared with the empty vector group, the random blood glucose levels at 12 weeks significantly increased in the over-expressed lncRNA H19 group (*P* < 0.05), while they decreased in the model, NC, and lncRNA H19-shRNA groups compared with the over-expressed lncRNA H19 group, and decreased in the lncRNA H19-shRNA group compared with the model and NC groups (*P* < 0.05). Compared to the basal blood glucose levels, the blood glucose levels after modeling and random blood glucose levels at 12 weeks increased in the empty vector, over-expressed lncRNA H19, model, and NC groups (all *P* < 0.05). However, there was no significant difference in the basal level of blood glucose in the lncRNA H19-shRNA group (*P* > 0.05). Compared to the blood glucose levels after modeling, the random blood glucose at 12 weeks in the over-expressed lncRNA H19 group, the random blood glucose at 12 weeks significantly increased in the lncRNA H19-shRNA, model and NC groups (*P* < 0.05), but decreased in the lncRNA H19-shRNA group (*P* < 0.05) (Table 1).

**Table 1:** Comparison of blood glucose (mmol/L) before and after the rat modeling in esch group (*n* = 10, mmol/L).

Group	Basal blood glucose	Blood glucose after modeling	Random blood glucose at 12 weeks
Normal group	6.00 ± 0.89	5.94 ± 0.92	6.29 ± 0.85
Model group	6.02 ± 0.85	21.99 ± 3.66^*a^	25.21 ± 3.24^*ab^
Empty vector group	5.84 ± 0.78	22.27 ± 3.52^*a^	25.46 ± 3.31^*ab^
Over-expressed lncRNA H19 group	6.00 ± 0.83	22.51 ± 3.67^*a^	28.79 ± 3.22^*#&ab^
NC group	6.17 ± 0.91	21.69 ± 3.51^*a^	25.15 ± 3.46^*ab^
LncRNA H19-shRNA group	6.15 ± 0.84	22.22 ± 3.68^*a^	6.31 ± 0.91^#$ab^

Notes: *, *P* < 0.05 as compared with the normal group; #, *P* < 0.05 as compared with the model group; &, *P* < 0.05 as compared with the empty vector group; $, *P* < 0.05 as compared to the NC group; a, *P* < 0.05 as compared with the basal blood glucose; b, *P* < 0.05 as compared with the blood glucose after the modeling; NC = negative control; lncRNA, long non-coding RNA; NC, negative group; shRNA, short hairpin RNA.

There was no significant difference in body weight before and after modeling in each group (all *P* > 0.05). As compared with the normal group, the body weight at 12 weeks decreased in the empty vector, over-expressed lncRNA H19, model, and NC groups, but did not change in the lncRNA H19-shRNA group (*P* > 0.05). Compared to the empty vector group, the body weight at 12 weeks was significantly reduced in the over-expressed lncRNA H19 group (*P* < 0.05), and increased in the model, NC and lncRNA H19-shRNA groups when compared with the over-expressed lncRNA H19 group (*P* < 0.05). The body weight at 12 weeks significantly increased in the lncRNA H19-shRNA group compared with the model and NC groups (*P* < 0.05), and there was no statistically significant difference between these two groups (*P* > 0.05). Compared with the basal body weight and the body weight after the modeling, the body weight at 12 weeks significantly decreased in the empty vector, over-expressed lncRNA H19, model and NC groups, while they increased in the lncRNA H19-shRNA group (all *P* < 0.05) (Table 2).

**Table 2:** Body weight (g) before and after the modeling in each group (mean ± s, *n* = 10).

Group	Basal body weight	Body weight after the modeling	Body weight at 12 weeks
Normal group	204.5 ± 5.3	207.4 ± 4.8	506.7 ± 13.8
Model group	209.0 ± 4.9	214.1 ± 4.1	473.5 ± 6.7^*ab^
Empty vector group	210.8 ± 3.7	206.9 ± 2.1	475.2 ± 5.4^*ab^
Over-expressed lncRNA H19 group	209.5 ± 3.7	212.8 ± 3.5	421.3 ± 3.9^*#&ab^
NC group	211.6 ± 3.8	208.5 ± 3.2	469.2 ± 4.3^*ab^
LncRNA H19-shRNA group	207.7 ± 8.3	213.1 ± 8.6	513.7 ± 4.8^#$ab^

Notes: *, *P* < 0.05 as compared with the normal group; #, *P* < 0.05 as compared with the model group; &, *P* < 0.05 as compared with the empty vector group; $, *P* < 0.05 as compared to the NC group; a, *P* < 0.05 as compared with the basal body weight; b, *P* < 0.05 as compared with the body weight after the modeling; lncRNA, long non-coding RNA; NC, negative group; shRNA, short hairpin RNA.

### Positioning navigation and space exploration abilities in DM rats

The positioning navigation and space exploration abilities of the rats were studied using the Morris water maze experiments. Compared with the normal group, the latency of positioning navigation significantly increased in the empty vector, over-expressed lncRNA H19, model, and NC groups, while the duration of space exploration significantly shortened (all *P* < 0.05). There was no significant difference between the lncRNA H19-shRNA and normal groups (*P* > 0.05). Compared with the model and empty vector groups, the latency of positioning navigation significantly prolonged, while the duration of space exploration significantly shortened in the over-expressed lncRNA H19 group (*P* < 0.05). There was no significant difference between the model and empty vector groups (*P* > 0.05), indicating that the learning and memory abilities of rats had a severe decline in the over-expressed lncRNA H19 group. Compared with the over-expressed lncRNA H19 group, the latency of positioning navigation decreased, and the duration of space exploration in the model, NC, and lncRNA H19-shRNA groups increased (*P* < 0.05). Compared with model and NC groups, the latency of positioning navigation in the lncRNA H19-shRNA group decreased, while the duration of space exploration increased (*P* < 0.05). There was no significant difference between the model and NC groups (*P* > 0.05). Together, these results suggest that the learning and memory abilities of the rats significantly improve in the lncRNA H19-shRNA group (Table 3).

**Table 3:** Positioning navigation and space exploration abilities of rats among six groups by Morris water maze experiment (*n* = 10).

Group	Positioning navigation (s)	Space exploration (s)
Normal group	20.10 ± 7.15	33.13 ± 5.17
Model group	34.25 ± 11.70^*^	24.55 ± 6.34^*^
Empty vector group	35.60 ± 9.90^*^	25.24 ± 5.53^*^
Over-expressed lncRNA H19 group	63.05 ± 8.30^*#&^	10.37 ± 4.18^*#&^
NC group	33.68 ± 11.47^*^	24.92 ± 5.17^*^
LncRNA H19-shRNA group	20.70 ± 7.02^$^	33.09 ± 4.35^$^

Notes: *, *P* < 0.05 as compared with the normal group; #, *P* < 0.05 as compared with the model group; &, *P* < 0.05 as compared with the empty vector group; $, *P* < 0.05 as compared to the NC group; lncRNA, long non-coding RNA; NC, negative group; shRNA, short hairpin RNA.

### Pathological changes of the hippocampal CA1 region in DM rats

The neuronal cells in the rat hippocampal CA1 regions were closely arranged; they were round and the nucleus and cytoplasm were clearly visible in the normal group. In the empty vector, over-expressed lncRNA H19, model, and NC groups, the neuronal cells were loosely arranged with changed morphology, including nuclear condensation and cytoplasm reduction, indicating apoptosis. In contrast, cell morphology in the lncRNA H19-shRNA group was similar to the normal group (Figure 3A). In the empty vector, over-expressed lncRNA H19, model and NC groups, the numbers of hippocampal neurons were significantly lower than in the normal group (*P* < 0.05), while there was no significant difference between the normal and lncRNA H19-shRNA groups (*P* > 0.05). Compared with the empty vector group, the numbers of hippocampal neurons in the over-expressed lncRNA H19 group (*P* < 0.05) decreased, suggesting that learning and memory in the over-expressed lncRNA H19 group decreased. On the other hand, learning and memory increased in the model, NC, and lncRNA H19-shRNA groups when compared with the over-expressed lncRNA H19 group (all *P* < 0.05). They also increased in the lncRNA H19-shRNA group when compared with the model and NC groups (*P* < 0.05); there was no significant difference between these two groups (*P* > 0.05). Together, these results indicate that learning and memory improved in the rat lncRNA H19-shRNA group (Figure 3B).

**Figure 3:** Pathological changes of hippocampal CA1 region of rats in each group and a number of neurons were couted using HE staining (×400) Notes: *, *P* < 0.05 as compared with the normal group; #, *P* < 0.05 as compared with the model group; &, *P* < 0.05 as compared with the empty vector group; $, *P* < 0.05 as compared to the NC group; NC = negative control, HE = Hematoxylin-eosin

### Electron microscopy of the hippocampal CA1 region in DM rats

The ultrastructural changes of the hippocampal CA1 neurons were mainly manifested as the synaptic changes. Compared with the normal group, the number of synaptosomes in the empty vector group, the over-expressed lncRNA H19 group, the model group and the NC group decreased, while their synaptic degeneration gap increased with a progress of mitochondrial vacuolization inside the synapses. In addition, the depth of condensed matters in synaptosomes was decreased after contacting the synapses. In the lncRNA H19-shRNA group, the ultrastructures were similar to those in the normal group (Figure 4A).

**Figure 4:** Ultrastructures of hippocampal CA1 region of rats in each group were observed by an electron microscope (×400) Notes: **A.**, Electron microscopic images of the ultrastructures in the hippocampal CA1 region of the rats in each group; **B.**, Statistics of synaptosomes in each group of rats; *, *P* < 0.05 as compared with the normal group; #, *P* < 0.05 as compared with the model group; &, *P* < 0.05 as compared with the empty vector group; $, *P* < 0.05 as compared to the NC group; NC = negative control.

Compared to the normal group, the number of synaptosomes in the empty vector group, the over-expressed lncRNA H19 group, the model group and the NC group decreased (*P* < 0.05), while there was no significant difference between the lncRNA H19-shRNA group and the normal group (*P* > 0.05). Compared with the empty vector group, the number of synaptosomes in the over-expressed lncRNA H19 group significantly decreased (*P* < 0.05). Compared with the over-expressed lncRNA H19 group, the number of synaptosomes in the model group, the NC group and the lncRNA H19-shRNA group increased (*P* < 0.05). Compared with the model and the NC groups, the number of synaptosomes in the lncRNA H19-shRNA group increased significantly (*P* < 0.05). There was no significant difference between the model and the NC groups (*P* > 0.05) (Figure 4B).

### Wnt signaling protein expression in the hippocampus of DM rats

Next, we analyzed gene and protein expression of the Wnt signaling pathway proteins in the hippocampus of rats among the six groups. Compared with the normal group, the expressions of Wnt3, β-catenin and TCF-1 was increased, while the expression of GSK-3β was decreased in the empty vector, over-expressed lncRNA H19, model, and NC groups (*P* < 0.05). There was no significant difference between the lncRNA H19-shRNA and normal groups (*P* > 0.05). In the over-expressed lncRNA H19 group, the expression of Wnt3, β-catenin, and TCF-1 was up-regulated while the expression of GSK-3β was down-regulated when compared to the empty vector group (*P* < 0.05). Compared with the over-expressed lncRNA H19 group, the expressions of Wnt3, β-catenin, and TCF-1 was reduced and the expression of GSK-3β was increased in the model, NC, and lncRNA H19-shRNA groups (*P* < 0.05). Compared to the model and NC groups, the expressions of Wnt3, β-catenin and TCF-1 was decreased, and the expression of GSK-3β was increased in the lncRNA H19-shRNA group (*P* < 0.05). There was no significant difference between the model and NC groups (Figure 5).

**Figure 5:** The expressions of Wnt signaling pathway-related proteins in the hippocampus of rats were measured by qRT-PCR and Western blotting Notes: **A.**, The expressions of Wnt signaling pathway-related proteins in the hippocampus of each group of rats were detected by Western blotting; **B.**, The quantification of the western-blotting; **C.**, The expressions of mRNA of Wnt signaling pathway-related proteins in the hippocampus of rats in each group were detected by qRT-PCR; *, *P* < 0.05 as compared with the normal group; #, *P* < 0.05 as compared with the model group; &, *P* < 0.05 as compared with the empty vector group; $, *P* < 0.05 as compared to the NC group; NC = negative control; qRT-PCR = quantitative real-time plymerace chain reaction.

### Apoptosis of hippocampal neurons in DM rats

We used TUNEL assay to evaluate apoptosis of hippocampal neurons of among the six groups of rats. The nuclei of normal hippocampal neurons were homogeneously blue-stained, and the nuclei of the late apoptotic cells were brown or dark brown. The nuclear pyknosis was irregular, and nuclear fragmentation and nuclear edge condensation could be seen under a high magnification lens. Compared with the normal group, the apoptosis rate of hippocampal neurons was increased in the empty vector, over-expressed lncRNA H19, model, and NC groups (*P* < 0.05), while there was no significant difference between the lncRNA H19-shRNA and normal groups (*P* > 0.05). Compared with the empty vector group, the apoptosis rate of hippocampal neurons was increased in the over-expressed lncRNA H19 group (*P* < 0.05), while it was decreased in the model, NC, and lncRNA H19-shRNA groups. There was no significant difference between the model and NC groups (*P* > 0.05) (Figure 6).

**Figure 6:** The apoptosis of hippocampal neurons of rats in each group was detected by TUNEL assay (×100) Notes: **A.**, The TUNEL staining images of rats in each group; **B.**, The statistics of apoptosis rates; *, *P* < 0.05 as compared with the normal group; #, *P* < 0.05 as compared with the model group; &, *P* < 0.05 as compared with the empty vector group; $, *P* < 0.05 as compared to the NC group; NC = negative control.

### Expression of apoptosis-related proteins in the hippocampus tissues of DM rats

Compared with the normal group, the protein levels of Bax, caspase-3, and caspase-8 were increased in the empty vector, over-expressed lncRNA H19, model, and NC groups, while the expression of Bcl-2 was decerased (*P* < 0.05). There was no significant difference between the lncRNA H19-shRNA and normal groups (*P* > 0.05). Compared to the empty vector group, the expression of Bax, caspase-3, and caspase-8 was increased, while the expression of Bcl-2 was reduced in the over-expressed lncRNA H19 group (*P* < 0.05). When compared with the over-expressed lncRNA H19 group, the expression of Bax, caspase-3, and caspase-8 was decreased and the expression of Bcl-2 was increased in the model, NC, and lncRNA H19-shRNA groups (*P* < 0.05). Compared with the model and NC groups, the expression of Bax, caspase-3 and caspase-8 was decreased in the lncRNA H19-shRNA group, while the expression of Bcl-2 was upregulated (*P* < 0.05). There was no significant difference between the model and NC groups (*P* > 0.05) (Figure 7).

**Figure 7:** The expressions of apoptosis-related proteins in the hippocampus tissues of rats in each group were detected by qRT-PCR and Western blotting Notes: **A.**, The expressions of apoptosis-related proteins in the hippocampus tissues of each group of rats were detected by Western blotting; **B.**, The quantification of the western-blotting; **C.**, The expressions of the mRNA of apoptosis-related proteins in the hippocampus tissues of each group of rats were detected by qRT-PCR; *, *P* < 0.05 as compared with the normal group; #, *P* < 0.05 as compared with the model group; &, *P* < 0.05 as compared with the empty vector group; $, *P* < 0.05 as compared to the NC group; NC = negative control; qRT-PCR = quantitative real-time plymerace chain reaction.

## DISCUSSION

Defects in hippocampal synaptic plasticity and disorders of memory and learning are the central nervous system complications of DM [15]. As cognitive impairment is mainly attributed to the hippocampal neuron loss [16], understanding the potential impact of lncRNA H19 on the apoptosis of hippocampal neurons *via* Wnt signaling may provide a theoretical foundation for the development of novel therapeutic strategies against the nervous system complications of DM.

Our present results demonstrate an increased expression of lncRNA H19 in rats with DM. LncRNA H19 is an imprinted gene at 90 kb 3’ of IGF2, regulating its expression and imprinting. Abnormal IGF2/H19 methylation has been associated with the development of intrauterine hyperglycemia [17]. In addition, DM induces DNA methylation alterations of H19 in the spermatozoa of rat offsprings [18].

Our study demonstrates a positive correlation between the expression of Wnt3 and β-catenin, and lncRNA H19 levels, suggesting that the Wnt signaling is activated by lncRNA H19. As a miRNA sponge, lncRNA H19 can attenuate the endogenous function of miR-22 and miR-141, both of which negatively correlate with the β-catenin expression, resulting in the activation of Wnt/β-catenin signaling [11]. Luo *et al* have demonstrated that H19 is associated with zeste homolog 2 (EZH2), and that the association can activate the Wnt/β-catenin signaling, thus providing another possible mechanism of the Wnt/β-catenin activation by lncRNA H19 [10]. Zhang *et al.* have confirmed this hypothesis and shown that H19 activates the Wnt signaling [19]. Additionally, the Wnt/β-catenin signaling pathway plays a major role in promoting the progression of malignant tumors, indicating that it regulates cell cycle and apoptosis [20]. The Wnt/β-catenin signaling activates HT-29-R cells, and H19 knockdown arrests the signaling in the parental cells [21]. Moreover, c-Myc and cyclin D1 are considered as genes of the Wnt/β-catenin signaling pathway, and knockdown of CUL4B promotes the cyclin D1- and c-Myc-regulated apoptosis in colorectal cancer cells [20]. In addition, miR-675-5p directly targets H19, and H19 enhances osteogenesis through activating the Wnt/β-catenin signaling pathway [11].

Our results demonstrate an increased expression of TCF-1, Bax and caspase 3, but decreased expression of GSK-3β and Bcl-2 in the empty vector, over-expressed lncRNA H19, model, and NC groups compared to the normal group, together with less hippocampal neurons and synaptosomes, and higher apoptosis rate of hippocampal neurons. The Wnt protein signals through a receptor complex, which is comprised of members of the Frizzled and low-density lipoprotein receptor-related protein families, and thus activates a variety of intracellular signaling pathways including the β-catenin/TCF signaling (known as the canonical Wnt signaling) [22]. Hence, activated Wnt signaling can increase the expression of TCF-1, a member of TCF family [23]. The canonical Wnt signaling has been showed to regulate both cell apoptosis and proliferation in a cell-context dependent manner, by which the activated Wnt/β-catenin signaling can not only enhance cell proliferation but also induce apoptosis in various cells [24]. An *in vitro* study has shown that the activation of Wnt/β-catenin signaling can also activate caspase 3 and decrease the mitochondrial membrane potential, resulting in the mitochondria apoptosis [25]. Wnt-induced apoptosis is also found in fibroblasts [26]. Wu *et al.* have found that activated Wnt signaling promotes macrophage apoptosis and up-regulates Bax and caspase-3, thus verifying our results [27]. The Wnt signaling pathway is activated by the binding of Wnt ligands to a receptor complex composed of a member of the Frizzled family and the low-density lipoprotein-receptor-related protein, which disrupts the regulatory complex of Adenomatous Polyposis Coli APC/Axin/GSK-3β by activating cytoplasmic adaptor protein disheveled phosphorylation [27]. In addition, another study has demonstrated that activation of Wnt signaling inactivates GSK-3β, leading to dephosphorylation and stabilization of β-catenin in the cytosol [28]. MiRNAs, such as miR-675, also regulate lncRNAs in glioma [29]. Furthermore, overexpression of lncRNA H19 promotes the proliferation of T/G HA-VSMC in miR-675 *in vitro* [30].

Finally, prolonged latency of place navigation and the shorter duration of spatial exploration were observed in the over-expressed lncRNA H19, model, and NC groups compared with the normal group, whereas the lncRNA H19-shRNA group exhibited the opposite results. As lncRNA H19 promotes apoptosis of hippocampal neurons and synaptosomes *via* Wnt signaling, silencing lncRNA H19 could increase the survival of hippocampal neurons. Newborn neurons may be involved in hippocampal functions particularly dependent on the dentate gyrus, such as pattern separation, which may also make distinct contributions to learning and memory [31]. Stranahan *et al* have conducted a study focused on Morris water maze and shown that spatial memory is impaired in DM rats along with decreased hippocampal neurogenesis [3].

Together, our results demonstrate that lncRNA H19 is highly expressed in rats with DM, resulting in activated Wnt signaling and increased apoptosis of hippocampal neurons. However, in rats in the lncRNA H19-shRNA group, apoptosis of hippocampal neurons is effectively suppressed, indicating that inhibition of lncRNA H19 may be a promising method for treatment of cognitive decline of patients with DM. However, further studies are needed to explore how the Wnt signaling can both enhance cell proliferation and induce apoptosis in hippocampal neurons.

## MATERIALS AND METHODS

### Ethics statement

The animal experiments were approved by the ethics committee of the First Hospital of Jilin University. All animal experiments followed the guidelines of the Management and Use of Laboratory Animals published by the National Institutes of Health.

### Animal model

Sixty male SD rats that were 8 weeks old and weighed 180-220 g, were purchased from Shanghai Laboratory Animal Center (SLAC), Shanghai, China. The rats were kept in a clean animal facility with constant humidity and temperature. After one week of adaptation, 50 rats were assigned into a DM group, and the other 10 rats were assigned into a control group with no intervention. The DM rat model was induced by a single injection of a streptozotocin (STZ) solution (Sigma-Aldrich Chemical Company, St Louis MO, USA) at a dose of 70 mg/kg of body weight. STZ was dissolved in a sodium citrate buffer, pH 4.5, at 0.1 mmol/L concentration. One day before the DM induction, the rats fasted for more than 8 h, but water drinking was allowed. After STZ injection, venous blood from rat tails was collected. When the glucose concentration was over 18 mmol/l, the DM model was considered successful, but the rats were not used if their blood glucose levels did not reach the requirement.

### Over-expression of lncRNA H19-short hairpin RNA (shRNA) or knock down of the source of lncRNA H19 lentivirus particles

The plasmid and lentiviral packaging system in the over-expressed lncRNA H19 group and empty vector group were provided from Thermo Scientific Open Biosystems. The high titer lentiviral particles in the over-expressed lncRNA H19 group were constructed, packaged, and concentrated by our laboratory, which was determined by 1 × 10^10^ TU/ml final concentration for brain injection. LncRNA H19-shRNA is a GIPZ lentiviral vector carrying the monoclonal small fragment shRNA directed against rats. The negative control group (NC) was a nonsense sequence. Both shRNA plasmids and lentiviral packaging system were purchased from Thermo Scientific Open Biosystems. Prior to the experiment, 8% glycerol was used as the organic solvent to purify and collect the virus with a titer not less than 1 × 10^10^ TU/ml, and the final titer for brain injection was 1 × 10^10^ TU/ml.

### Animal grouping

Animals were divided into 6 groups (*n* = 10 in each group): normal group (normal rats), model group (DM rats), empty vector group (DM rats receiving empty vectors), over-expressed lncRNA H19 group (DM rats injected with lncRNA H19 over-expression lentiviral particles), NC group (DM rats injected with nonsense vectors) and lncRNA H19-shRNA group (DM rats injected with lncRNA H19-shRNA lentiviral vectors).

### Stereotactic injection

After successful establishment of the DM model and stabilization of blood glucose, the hippocampal CA1 region was selected as the injection point, and the brain injection was conducted for each animal group. The rats were anesthetized with intra-peritoneal injection of 1% glutaraldehyde solution at a dose of 40 mg/kg, and their heads were fixed on a stereotaxic apparatus. The injection coordinates were in reference to the rat brain mapping map [32]: 3.5 ∼ 4 mm behind anterior fontanel, incision at ± 2.8 ∼ 3 mm beside the midline, and skull dorsal depth of -2.8 ∼ -3.0 mm. In the over-expressed lncRNA H19 group, 5 μl of lncRNA H19 over-expression lentiviral particles at same viral titer were injected at both sides. In the lncRNA H19-shRNA group, 5 μl of lncRNA H19-shRNA lentiviral particles [the overall length of H19 (NR_002196), interfere sequence: CGTGACAAGCAGGACATGA] in equal viral titer were injected at both sides. In the NC group, 5 μl of viral particles carrying nonsense sequences were injected at both sides with the same viral titer. Blood glucose and body weight of all rats were monitored during the experiment. Rats in all groups were sacrificed 12 weeks after injection, and whole brain tissues were used for further experiments.

### Morris water maze test

The learning and memory abilities of the rats were evaluated by an animal behavioral learning and memory system (Viewpoint Life Sciences, Lyon, France). Before the experiment, adequate amount of water was filled in the water maze, and skim milk powder was used to adjust the light. To minimize errors, experiments were carried out at the same time with the same water temperature. During the first 4 days, positioning navigation experiments were carried out. The rats were placed in water facing the walls, and the rats that climbed onto the platform were observed and recorded by the camera for 1 min. The rats would be manually guided to the platform and stayed there for 30 s, if they still could not climb onto the platform after 1 min, and the latency period was recorded as 1 min. The learning ability of rats in each group was mainly manifested as the latency period in the first 4 days. Space exploration experiments were carried out in the fifth day: the platform was withdrawn, and the rats were placed into the water from the B quadrant. The results of the memory capacity was the swimming time in the D quadrant during a 1-min period.

### Hematoxylin-eosin (HE) staining and cell counting

After blood collection, whole brain tissues were quickly removed and placed on a glacial table, washed with saline, fixed in 4% formaldehyde solution, embedded with paraffin, and sliced. The tissues were then stained with HE for 5 min, differentiated, washed, stained again with HE, dehydrated with gradient alcohol, and mounted with a neutral gum in order to be observed under an inverted microscope. The cell count of hippocampal neuron was centered at the junction of the hippocampal CA1 region and the extension line from the end of the upper and lower branches in the dentate gyrus of the hippocampal tissue. Centered at this junction, and extended to both directions by 0.5 mm, a 1 mm length was chosen as the experimental count range for the cells in the hippocampal CA1 region. The cells were counted and photographed.

### Electron microscopy

After blood collection, whole brain tissues were placed on a glacial table, washed with saline, and fixed with 2.5% glutaraldehyde solution. The hippocampus tissues were dissected under an inverted microscope. Tissue sections of 1 mm^3^ in the hippocampal CA1 region were fixed with 2.5% glutaraldehyde solution, washed with phosphate buffered saline (PBS), dehydrated, embedded, sliced, and stained with lead citrate and acetic acid. The ultrastructure of synaptosomes and surrounding organelles in hippocampal CA1 region was observed under an electron microscope. The number of synaptosomes was counted and analyzed by the Physical Disector (Disector Countor 1.0) software.

### Western blotting

Tissue proteins were extracted and their concentration was determined using a BCA kit (Wuhan Boster Biological Technology Ltd., Wuhan, Hubei, China). The protein extracts were boiled in a sample buffer for 10 min, separated on a 10% polyacrylamide gel, and transferred to PVDF membrane. The membranes were blocked with 5% bovine serum albumin (1 h, RT), and incubated with primary antibodies (Cell Signaling Technology) for Wnt3 (1:1000 dilution, #9248), GSK-3β (1:1000 dilution, #8240), glyceraldehyde phosphate dehydrogenase (GAPDH) (1:500 dilution, #5174), and β-catenin (1:1000 dilution, #9566). In addition, antibodies against TCF-1 (1:1000 dilution, sc-79542), Bax (1:1000 dilution, sc-23959), Bcl-2 (1:1000 dilution, sc-7382), caspase-3 (1:1000 dilution, sc-65496), and caspase-8 (1:1000 dilution, sc-81656) purchased from Santa Cruz Biotechnology were used. The membranes were then washed in TBST and incubated with corresponding secondary antibodies (1 h, RT). GAPDH was used as an internal reference. Bio-Rad Gel DOC EZ imager was used to develop the membranes. The images were evaluated using the Image J software.

### Quantitative real-time polymerase chain reaction (qRT-PCR)

Total RNA was extracted and reverse transcription of cDNA were performed according to the kit instructions (QIAGEN, Valencia, CA). Primers were designed using the Primer 5.0 primer design software according to the gene sequences published in the Genbank database. The primers (Table 4) were synthesized by Shanghai Sangon Biological Engineering Technology & Services Co., Ltd. (Shanghai, China). The reaction system of PCR was 20 μl: 10 μl of SYBR PremixExTaq, 0.8 μl of forward and reverse primers, 0.4 μl of ROX Reference Dye II, 2 μl of DNA template, and 6.0 μl of dH_2_O. The reaction conditions were as follows: pre-denaturation at 95°C for 30 s, 40 cycles of denaturation at 95°C for 5 s, annealing at 60°C for 30 s, and extension at 72°C for 30 s. The internal control used in our study was GAPDH. The relative expression of the target gene was calculated as 2^-△△^Ct, wherein Ct value is the cycle threshold [33].

**Table 4:** Primer sequence for qRT-PCR.

Gene	Forward primers (5’-3’)	Reverse primers (5’-3’)
LncRNA H19	TACAACCACTGCACTACCTG	TGGAATGCTTGAAGGCTGCT
Wnt3	GCCTCTGACAAGCCCGAAA	GCGACGCCCCCAATAGTT
GSK-3β	GGCTGTGTGTTGGCTGAAT	GATTGCCTCTGGTGGAGTTC
β-catenin	GCTGATTTGATGGAGTTGGA	TCAGCTACTTGTTCTTGAGTGAA
TCF-1	TGGCTTCTACTCCCTGACC	CTGCCTTGGACTCTGCTT
Bax	AAGCTGAGCGAGTGTCTCAAG	CAAAGTAGAAAAGGGCGACAAC
Bcl-2	CGCATCAGGAAGGCTAGAGTT	CAGACATTCGGAGACCACACT
Caspase-3	GAGCACTGGAATGTCATCTCGCTCTG	TACAGGAAGTCAGCCTCCACCGGTATC
Caspase-8	TGCCCTCAAGTTCCTGTGCTTGGA	GGATGCTAAGAATG-TCATCTCC
GAPDH	ACCACAGTCCATGCCATCAC	TCCACCACCCTGTTGCTGTA

Note: qRT-PCR, quantitative real-time polymerace chain reaction.

### TUNEL staining

TUNEL detection kit (F. Hoffmann-La Roche Ltd., Basel, Switzerland) was used to detect the apoptosis. The hippocampus tissues were fixed for 30 min at room temperature, rinsed with PBS, and immersed in 0.2% Triton X-100 solution for 5 min to enhance the permeability. Subsequently, the samples were washed with PBS and dried, and 50 μl of reaction mixture (ratio of concentrated enzyme solution and labeling solution was 1: 9) were added. The samples were washed with PBS and observed under a fluorescence microscope. In each slide, 5 view fields were randomly selected and the number of apoptotic cells was counted as the apoptotic rate = the number of apoptotic cells / total cells × 100%.

### Whole genome methylation and detection of H19 promoter region

DNA from the hippocampal tissues was extracted, and methylation was analyzed using the whole gene methylation kit.

The pyrophosphate sequencing was used to detect DNA methylation in DMR region two locus of Lnc RNA H19. The primers used for sequencing were synthesized (Qiagen, Hilden, Germany). DNA from 100 ng pyrophosphate was amplified using a reaction system that included 5×PCR buffer, 10 mM dNTP, 50 mM upstream and downstream primers, and 1 U DNA polymerase. The PCR conditions were: 95°C for 3 min, cycled 40 times at 95°C for 30s, annealed at 60°C for 30s and 72°C for 1 min, and finally at 72°C for 7 min. The sequencing program of PCR product was tested using Pyromark Q96 ID. The methylation was analyzed using the Allele quantitative software. All samples was measured 3 times.

### Statistical analysis

Data were analyzed using the SPSS18.0 statistical software, and the results were expressed as mean ± s. The comparisons between two groups with normal distributions were detected using the *t* test. The comparisons among multiple groups were detected by One-Way analysis of variance (ANOVA), and *P* < 0.05 indicated a statistically significant difference.
